RETRACTED

# Akt Regulates Drug-Induced Cell Death through Bcl-w Downregulation

**DOI:** 10.1371/journal.pone.0004070

**Published:** 2008-12-30

**Authors:** Michela Garofalo, Cristina Quintavalle, Ciro Zanca, Assunta De Rienzo, Giulia Romano, Mario Acunzo, Loredana Puca, Mariarosaria Incoronato, Carlo M. Croce, Gerolama Condorelli

**Affiliations:** 1 Department of Cellular and Molecular Biology and Pathology, “Federico II” University of Naples, Naples, Italy; 2 Department of Molecular Virology, Immunology and Medical Genetics, Human Cancer Genetics Program, Comprehensive Cancer Center, The Ohio State University, Columbus, Ohio, United States of America; 3 IEOS, CNR, Naples, Italy; 4 Fondazione SDN, Naples, Italy; 5 IRGS, Biogem s.c.ar.l., Ariano Irpino (AV), Italy; 6 Facoltà di Scienze Biotecnologiche, “Federico II” University of Naples, Naples, Italy; University of Birmingham, United Kingdom

## Abstract

Akt is a serine threonine kinase with a major role in transducing survival signals and regulating proteins involved in apoptosis. To find new interactors of Akt involved in cell survival, we performed a two-hybrid screening in yeast using human full-length Akt c-DNA as bait and a murine c-DNA library as prey. Among the 80 clones obtained, two were identified as Bcl-w. Bcl-w is a member of the Bcl-2 family that is essential for the regulation of cellular survival, and that is up-regulated in different human tumors, such as gastric and colorectal carcinomas. Direct interaction of Bcl-w with Akt was confirmed by immunoprecipitation assays. Subsequently, we addressed the function of this interaction: by interfering with the activity or amount of Akt, we have demonstrated that Akt modulates the amount of Bcl-w protein. We have found that inhibition of Akt activity may promote apoptosis through the downregulation of Bcl-w protein and the consequential reduction in interaction of Bcl-w with pro-apoptotic members of the Bcl-2 family. Our data provide evidence that Bcl-w is a new member of the Akt pathway and that Akt may induce anti-apoptotic signals at least in part through the regulation of the amount and activity of Bcl-w.

## Introduction

Akt is a serine–threonine kinase downstream of PTEN/PI3K, involved in cellular survival pathways [1], [2]. In mammalian cells, the three Akt family members, Akt1/PKBα, Akt2/PKBβ, and Akt3/PKBγ are encoded by three different genes [3], [4]. They are ubiquitously expressed, although their levels are variable, depending upon the tissue type and pathological/physiological state. Increased expression or activation of Akt has been described as a frequent phenomena in human cancer [1], [5], [6]. Akt has been demonstrated to phosphorylate a number of proteins involved in apoptotic signaling cascades, including the Bcl-2 family member BAD [7], pro-caspase 9 [4], the forkhead transcription factors, FKHR and FKHRL1 [8], [9], and p21 cipWAF1. Phosphorylation of these proteins prevents apoptosis through several mechanisms [10]. Apoptosis, or programmed cell death, is an evolutionarily conserved mechanism of elimination of unwanted cells [11]. Apoptosis is triggered via two principal signaling pathways [12]. The extrinsic pathway is activated by the engagement of death receptors on the cell surface [13]. The other pathway is triggered by various intracellular and extracellular stresses, such as growth–factor withdrawal, hypoxia, DNA damage, and anticancer therapy [13], [14]. Intrinsic-pathway induced-apoptosis is generally regulated by the fine balance of Bcl-2 family proteins in a cell- and tissue-specific manner [11]. Apoptosis is believed to be the major mechanism responsible for chemotherapy-induced cell death in cancer. However, tumor cells often retain the ability to evade drug-induced death signals because of the activation of anti-apoptotic mechanisms [15]–[17]. Understanding these evading mechanisms is a first step needed for the design of rational anticancer therapy. Therefore, we decided to address the role of Akt in apoptosis resistance in human cancer by finding new partners involved in resistance to cell death. To this end, we performed a two hybrid screening in yeast using human full-length Akt c-DNA as bait and a murine c-DNA library as prey. Among the possible interactors of Akt, we decided to focus on Bcl-w, a member of the Bcl-2 family. Biochemical experiments confirmed the interaction of Akt with Bcl-w. Further, we demonstrate that Akt modulates the half-life of Bcl-w. We also found that Bcl-w is a substrate of Akt and, more importantly, that Akt regulates its anti-apoptotic activity and interaction with some of the pro-apoptotic members of the Bcl-2 family.

RETRACTED

## Methods

### Materials

Media, sera, and antibiotics for cell culture were from Life Technologies, Inc. (Grand Island, NY, USA). Protein electrophoresis reagents were from Bio-Rad (Richmond, VA, USA), and Western blotting and ECL reagents were from GE Healthcare. All other chemicals were from Sigma (St. Louis, MO, USA).

### Plasmids

Plasmids pEF FLAG(hs) Bcl-w , pEF EE Bax, pEF EE Bik, pEF EE Bad cDNAs were kindly provided by Elisabeth Cory and David Huang laboratories (Victoria, Australia). Akt wild type (HA-Akt, cDNA), Akt E40 K (constitutively active Akt cDNA, HA-Akt-D+) and Akt K179M (dominant negative Akt cDNA, HA-Akt-D-) were a kind gift of Prof. G.L. Condorelli (University of Rome “La Sapienza”).

### Cell culture

Human HeLa and HEK-293 cell lines were grown in DMEM containing 10% heat-inactivated FBS and with 2 mM L-glutamine and 100 U/ml penicillin-streptomycin.

### Yeast Two-hybrid System

All experiments were performed in the yeast reporter MaV203. The cDNA library was synthesized from rat FRTL-5 cell poly(A)^+^ RNA plasmid by Life Technologies and cloned into the pPC86GAL4AD vector, and was kindly provided by Prof. Roberto Di Lauro (Naples, Italy). Screening of the library was performed essentially following instructions for the ProQuest two-hybrid system (Life Technologies) and has been previously described [18]. The GAL4 DNA-binding domain/hAkt fusion was obtained from Dr. Alfonso Bellacosa (Fox Chase Cancer Centre, Philadelphia, Pennsylvania, USA). Subsequently, yeast pLEx4-Akt plasmid was transformed with the pPC86AD-cDNA library and plated onto plates lacking histidine in the presence of 3AT (aminotriazole; 10 mM). Approximately 1.2×10^6^ individual clones were plated, and about 200 grew on the selective medium. Resistant colonies were grown on a master plate and then replica-plated onto selection plates to determine their ability to induce three independent reporters (*HIS3*, *URA3*, and *lacZ*). Eighty independent clones were isolated after this first screening. DNA was isolated from each positive clone and sequenced to identify the inserts. Independent pPC86AD clones were retransformed into yeast and tested for interaction with a fresh Akt clone.

### Generation of Bcl-w deletion mutants

We generated by PCR two deletion mutants of Bcl-w cDNA, using as template the plasmid pEF FLAG Bcl-w: the following primers were used for the bclw-BH4 mutant, which included only the N-terminal BH4 domain (45 aa): BH4-For-HINDIII:cccaagcttatggactacaaagacgatgacgataaag and BH4-Rev-Xba1: gctctagaggcttggtgcagcgggtc; the following primers were used for CT-Bcl-w, which included the remaining coding sequence of 97aa: CT-For-HINDIII: cccaagcttcccagcagctgacccgct and CT-Rev-Xba1: gctctagatcacttgctagcaaaaaaggccc.

Temperature cycles were the following: 95°C 1 minute; 95°C 50 seconds, 60°C 50 seconds, 68°C 7 minutes for 35 cycles; 68°C 2 minutes. The amplified sequences were cloned in p3X-Flag-CMV previously linearized with the restriction enzymes HINDIII and XbaI.

### Generation of stable transfectants

HeLa cells were transfected with 4 µg of Flag-Bcl-w cDNA using lipofectamine 2000 according to the manufacturer's protocol (InVitrogen, Carlsbad, CA). After 48 hr of transfection, cells were selected using a medium containing 10% FBS, 2 mMol L-glutammine, 100 U/ml pen/strep, and 3.75 µg/ml of puromicine. After 15 days the clones were isolated and maintained in culture with 2.5 µg/ml of puromicine. Twenty colonies were isolated and tested through western blot to verify the expression of the construct.

RETRACTED

### Western blotting

Total protein from HeLa and HEK 293 cells was extracted with RIPA buffer (0.15 mM NaCl, 0.05 mM Tris-HCl, pH 7.5, 1% Triton, 0.1% SDS, 0.1% sodium deoxycolate and 1% Nonidet P40). Fifty µg of sample extract were resolved on 7.5–12% SDS-polyacrylamide gels using a mini-gel apparatus (Bio-Rad Laboratories, Richmond, CA) and transferred to Hybond-C extra nitrocellulose. Membranes were blocked for 1 hr with 5% non-fat dry milk in TBS containing 0.05% Tween-20, incubated over night with primary antibody, washed and incubated with secondary antibody, and visualized by chemiluminescence. The following primary antibodies were used: Anti Flag M2 and anti-β-actin antibody from Sigma (St. Louis, MO, USA), anti HA and anti EE from Covance (Berkeley,CA USA); anti Bcl-w from Abcam (Cambridge, MA); anti-Akt, -Phospho Akt substrate, -phospho ser473 Akt from Cell signalling (Danvers, MA USA); anti-Bcl2, - BAD, -BIK and -BAX from Santa Cruz, Inc (Santa Cruz, CA USA), caspase -9 and -3 from Cell Signaling (Danvers, MA USA), and PARP antibodies from Santa Cruz (Santa Cruz, CA USA).

### Phosphorylation experiments

In order to study Bcl-w phosphorylation in intact cells, 293 cells were transiently transfected with different Akt cDNAs constructs as indicated. After 24 h, the cells were rinsed with 150 mM NaCl and incubated in serum-free culture medium for 16 h at 37°C. Insulin (final concentration, 100 nM) or 20% serum was then added, and the cells were rapidly rinsed with ice-cold saline followed by solubilization with 0.5 ml of RIPA buffer per dish for 1 hr at 4°C. Lysates were centrifuged at 5,000×g for 20 min, and solubilized proteins were precipitated with the indicated antibodies, separated by SDS-PAGE, and revealed by western blot with the anti-Akt substrate antibody that recognizes all the phosphorylated Akt substrates (Cell Signaling, Danvers, MA USA). Phospho-(Ser/Thr) Akt Substrate Antibody preferentially recognizes peptides and proteins containing phospho-Ser/Thr preceded by Lys/Arg at positions −5 and −3. Some cross-reactivity has been described for peptides that contain phospho-Ser/Thr preceded by Arg/Lys at positions −3 and −2, thus recognizing also a low-stringency Akt kinase motif.

### Immunoprecipitation

Cells were cultured at a final concentration of 90% in p100 plates. The cells were harvested with RIPA Buffer on a shaker for 30 minutes. 1 mg of total extract was immunoprecipitated using the indicated antibodies (5 µg/ml Anti-FLAG, 2 µg/ml Anti-HA, 3 µg/ml anti-Akt, 5 µg/ml anti-Bcl-w, 3 µg/ml anti-EE), for 16 hrs on shaker. Then, A/G beads (Santa Cruz, Santa Cruz, CA USA) were added for two hrs. The beads were washed for three times with washing buffer (50 mM Tris Hcl pH 7.5, 150 mM NaCl, 0.1% Triton, 10% glycerol), and then 20 µl of sample buffer was added; the samples were boiled at 100°C for 5 minutes and then the supernatants resolved by SDS-PAGE.

RETRACTED

### Cytosol/mitochondria separation

Cells were grown in p100 plates and the mitochondrial and cytoplasmic fractions isolated using the Mitochondria/Cytosol Fractionation Kit (Biovision San Francisco, CA USA) according to the manufacturer's protocol.

### Akt Kinase Assay

Akt activity was assayed in vitro as previously reported [19]. Briefly, HEK-293 cells were transfected with 4 µg of Flag-Bcl-w cDNA. 1 mg of total cell extract was immunoprecipitated using an anti-FLAG antibody (Sigma) and A/G beads (SantaCruz, Santa Cruz, CA USA) for 18 hr. The beads were incubated in a kinase reaction mixture containing 20 mM HEPES [pH 7.2], 1 mM MgCl_2_, 10 mM MnCl_2_,1 mM dithiothreitol, 5 mM ATP, 0.2 mM EGTA, 1 mM protein kinase inhibitor, 10 µCi of [γ–^32^P]ATP, and 2 µg of rAkt (Cell signaling, Danvers, MA USA) for 30 minutes at room temperature. The samples were boiled at 100°C for 5 minutes, centrifuged and the supernatant loaded on a 12.5% maxi protean gel (BioRad, Richmond VA, USA). The gel was run overnight and then visualized by autoradiography.

### Cell death and cell proliferation quantification

Cells were plated in 96-well plates in triplicate and incubated at 37°C in a 5%CO_2_ incubator. Different chemotherapics (30 mg/ml cisplatin, 10 mg/ml epirubicin) were added for 24 hrs to the medium. Cell viability was evaluated with the CellTiter 96® Aqueous One Solution Cell Proliferation Assay (Promega, Madison, WI), according to the manufacturer's protocol. Metabolically active cells were detected by adding 20 µl of MTT to each well. After 2 h of incubation, the plates were analyzed in a Multilabel Counter (Bio-Rad, Richmond, VA, USA). Apoptosis was assessed using PI (propidium iodide)-FITC staining followed by flow cytometric analysis. Cells were seeded at 1.8×10^6^ cells per 100 mm dish, grown overnight in 10% FBS/DMEM, washed with PBS, then treated for 24 hours with chemotherapics. Following incubation, cells were washed with cold PBS and removed from the plates by mild trypsinization. The resuspended cells were washed with cold PBS and stained with PI-FITC staining according to the instructions provided by the manufacturer (Roche Applied Science, Indianapolis, IN). Cells (50,000 per sample) were then subjected to flow cytometric analysis. Flow cytometry analysis were done as described [20]. The percentage of apoptosis indicated was corrected for background levels found in the corresponding untreated controls.

RETRACTED

### siRNA transfection

HeLa cells were cultured to 80% confluence and transiently transfected using LIPOFECTAMINE 2000 with 100 nM anti-Akt siRNA (Dharmacon, Lafayette, CO USA), a pool of 4 target-specific 20–25 nt siRNAs, or 150 nM anti-Bcl-w si-RNA (InVitrogen, Carlsbad, CA) with 6 µl transfection reagent, as described in the manufacturer's protocol.

## Results

### Akt interacts with Bcl-w

To find new interactors of Akt, we performed a yeast two-hybrid screening with human full-length Akt c-DNA sequence as bait and a murine c-DNA thyroid library as prey. Among the 100 clones obtained, two were identified as Bcl-w, covering its full coding sequence. To confirm the interaction between Akt and Bcl-w, we immunoprecipitated proteins from untreated, Akt-transfected, and Bcl-w-transfected cells with an anti-Bcl-w antibody. We found that Akt co-immunoprecipitates with Bcl-w in extracts from untransfected and transfected cells (Figure 1A and 1B). The extent of Akt binding with Bcl-w was comparable to that with its substrate, Bad (Figure 1B).

**Figure 1:** Akt interacts with Bcl-w. (A) Co-immunoprecipitation of endogenous Akt with Bcl-w. Wt HeLa cells were lysed and 1 mg of protein extract immunoprecipitated using an anti-Bcl-w antibody. Immunoprecipitates and total lysates (50 µg) were separated on 12%SDS polyacrilamide gel and blotted with an anti-Akt antibody. As negative control, proteins were incubated with beads without antibody (B) Co-immunoprecipitation of transfected Akt with FLAG-Bcl-w or EE-BAD. HEK-293 cells were tansfected with 2 µg of HA-Akt and 2 µg of FLAG-Bcl-w or EE-BAD cDNAs, as indicated. After 48 hr, cells were lysed, and 1 mg of protein extract was immunoprecipitated using an anti-HA antibody. Immunoprecipitates were subsequently blotted with anti-HA, anti-Flag or anti-EE antibodies, as indicated. (C) HEK-293 cells were transfected with 2 µg of either wt-Bcl-w cDNA or the deletion mutants, Bcl-w/BH4 or Bcl-w/CT, as indicated. Protein extracts were immunoprecipitated using an anti-Akt antibody. Immunoprecipitates and total lysates were resolved on 12%SDS-PAGE and transferred to Hybond-C nitrocellulose. Membranes were incubated with an anti-FLAG antibody. Both deletion mutants, Bclw/BH4 and Bclw/CT, immunoprecipitated with Akt.

Bcl-w contains four Bcl-2 homology (BH) domains and a transmembrane (TM) fragment at the C-terminal region, important for its insertion into the mitochondrial outer membrane. We verified whether these regions are important for the interaction with Akt. For this, HA-Akt cDNA was transfected together with one of two Bcl-w domain-region cDNAs obtained by PCR and fused to the FLAG epitope: these were the BH4 domain (45 aa) of Bcl-w, located at the N-terminus, and the remaining portion of the protein (97aa). Extracts were immunoprecipitated with an anti-Flag antibody and blotted with an anti-HA antibody. We found that Akt interacts with both Bcl-w deletion mutants, indicating that Akt may interact with Bcl-w at multiple sites (Figure 1C).

RETRACTED

### Role of Akt activation on Akt/Bcl-w interaction

To find whether the activity of Akt influences its interaction with Bcl-w, HeLa cells were transfected either with wild type Akt (Akt wt) cDNA or with one of two mutants: an HA-tagged kinase dead-Akt construct (Akt D−) with dominant negative functions, and a constitutively active Akt construct (Akt D+). Protein extracts were immunoprecipitated with a monoclonal anti-HA antibody and then blotted with an anti-FLAG antibody. We found that Bcl-w interacts with wild type Akt and more efficiently with the activated kinase, but not with the kinase-dead Akt (Figure 2A).

**Figure 2:** Akt activity regulates Bcl-w expression. (A) HeLa cells were transfected with 2 µg of HA-Akt wt, Akt D+, or HA-Akt D− cDNA and 2 µg Flag-Bcl-w for 48 hrs. Protein extracts were immunoprecipitated with an anti-HA monoclonal antibody. Immunoprecipitates were resolved on 12% SDS-PAGE and transferred to Hybond-C nitrocellulose. Membranes were incubated with anti-Flag antibody (0.2 µg/ml). 50 µg of total sample extracts were also analyzed by western blot using the indicated antibodies. Loading control was obtained using anti-β actin antibody. (B) HeLa cells were transfected with 4 µg of HA-Akt wt, HA-Akt D+, or HA-Akt D− cDNA for 48 hrs. Protein extracts were blotted with anti-Bcl-w antibody in order to detect endogenous levels of Bcl-w. Loading control was obtained with anti-β actin antibody. (C) Cells were transfected with 100 nM of siAkt-RNA for 48 hrs. Cellular proteins were solubilized and analyzed by western blot using the indicated antibodies. (D) HeLa cells were treated with 10, 20 or 40 µM of LY294002 for 24 hrs. Protein extracts were analyzed by western blot using the indicated antibodies. Loading control was obtained using anti-β actin antibody. (E) Bcl-w HeLa cells were treated with 10 µM of MG-132 for 8 hrs. 40 µg of protein extracts were analyzed by western blot with anti-Bcl-w antibodies. Loading control was obtained using anti-β actin antibody.

### Akt regulates Bcl-w expression

When we transfected cells with Akt D−, we noticed a fall in the expression of Bcl-w (Figure 2A). Therefore, lack of interaction between Bcl-w and the kinase-dead Akt could have been due to reduced expression of Bcl-w rather than to poor interaction with Akt D−. To address this issue, we inhibited Akt in three different ways: by interfering with its endogenous function; by treating cells with Akt-siRNA; and by inhibiting the PI3K/Akt pathway with a specific drug. In order to interfere with endogenous Akt activity, we transfected cells with the previously described Akt mutant cDNAs (Akt wt, Akt D+, and Akt D−). We found that Bcl-w was reduced after transfection with inactive Akt, whereas Bcl-w expression increased upon transfection with Akt D+ (Figure 2B). In order to knock down endogenous Akt, HeLa cells were transfected with a pool of Akt siRNAs. We found that endogenous Akt expression, analyzed by Western blot, was reduced by >80% after 48 hrs. This reduction in Akt expression was followed by a drastic reduction in the level of Bcl-w. Moreover, the expression of the anti-apoptotic protein, Bcl-2, but not of the pro-apoptotic protein, Bax, was also reduced (Figure 2C). Finally, incubation of HeLa cells with 10, 20 or 40 µM of LY294002, a specific inhibitor of the PI3K pathway, resulted in reduced amount of Bcl-w protein (Figure 2D). All these results provide evidence that the kinase activity of Akt regulates the expression of Bcl-w.

RETRACTED

To gain insight on the mechanism of Akt-mediated Bcl-w regulation, we treated Bcl-w/HeLa cells with the proteasome inhibitor, MG-132, for 8 hrs and then analyzed Bcl-w levels by western blot (Figure 2E). The inhibition of the proteasome did not result in an increase in Bcl-w expression, suggesting that the ubiquitin pathway is not directly involved in the regulation of Bcl-w by Akt.

### Role of Akt in Bcl-w subcellular localization

Bcl-w is an anti-apoptotic protein weakly linked to the outer mitochondrial membrane [21]. To verify its intracellular localization, extracts of HeLa cells were fractionated to isolate mitochondria from the cytosol. We found that Bcl-w is present mainly in mitochondrial protein extracts (Figure 3A). To clarify the role of Akt in determining Bcl-w cellular localization, HeLa cells were transfected with Akt wt, Akt D+, or Akt D− cDNAs before fractional separation. We found that the presence of the kinase-dead Akt mutant reduced the amount of Bcl-w linked to the mitochondrial fraction and induced only a slight increase in the cytosolic one (Figure 3B). Similar results were obtained in cells transfected with Akt siRNA (Figure 3C). Thus, Akt acts mainly on Bcl-w expression.

**Figure 3:** Akt controls Bcl-w localization. (A) HeLa cells were subjected to fractionated separation of mitochondrial/cytosolic proteins using a mitochondria/cytosol fractionation kit (Biovision). Protein extracts were loaded onto 15% SDS polyacrilamide gel, and analyzed by western blot by anti-Bcl-w antibody. As a control of the mitochondrial fraction, an anti-cox4 antibody was used. (B) HeLa cells were transfected with 2 µg of HA-Akt WT, D+, or D− for 48 hrs. Cells were subjected to mitochondria/cytosol separation as above. Protein extracts were analyzed by western blot using anti-Bcl-w, anti-Akt, or anti-cox4 antibodies. (C) Cells were transfected with 100 nM of siAkt-RNA for 48 hrs. Cytosol and mitochondria were isolated as described in the methods and analyzed by western blot using the indicated antibodies.

RETRACTED

### Akt phosphorylates Bcl-w

Akt is a serine threonine kinase that phosphorylates different pro- and anti-apoptotic proteins. Thus, in vitro and in vivo phosphorylation assays were performed to uncover whether Bcl-w is a substrate of Akt. For in vitro assays, cells were transfected with Flag-Bcl-w and the extracts obtained immunoprecipitated using a monoclonal anti-Flag antibody. Immunoprecipitates were incubated with a constitutively active Akt recombinant protein in the presence of γP^32^ATP. We found that Akt phosphorylates Bcl-w in vitro, although not with the same efficiency as histone H2B (Figure 4A).

**Figure 4:** Akt phosphorylates Bcl-w in vitro and in vivo. (A) HeLa cells were transfected with 2 µg of DNA of Flag Bcl-w, solubilized, and 1 mg of protein extract was immunoprecipitated with an anti-M2 Flag antibody. Immunoprecipitates were incubated with recombinant constitutive active Akt (rAkt), and in vitro kinase assay was conducted as described in the methods. Samples were loaded onto 2.5% SDS-PAGE and analyzed by autoradiography. As positive control we used Histone2B (H2B). (B) HeLa Bcl-w stable expressing clones were serum starved for 18 hrs and then stimulated with 100 nM insulin or with 20% serum for 15 min as indicated. Cells were solubilized and immunoprecipitated with an anti-M2 Flag antibody. Immunoprecipitates were loaded onto SDS-PAGE and blotted with an anti-phospho Akt substrate antibody that recognizes all the phosphorylated Akt substrates. Total extracts were analyzed by western blot using the indicated antibodies. (C) HeLa cells were transfected with 2 µg of pcDNA3 empty vector or 2 µg of HA-GSK3β, and 2 µg of Flag-Bcl-w for 48 hrs. Cells were stimulated with 100 nM insulin for 15 min, solubilized, immunoprecipitated using an anti-HA antibody, and analyzed by western blot using an anti-phospho-Gsk3 antibody. Total extracts were analyzed by western blot using the indicated antibodies. Bcl-w overexpression does not affect Akt activity.

To study the effects of Akt kinase activity on Bcl-w phosphorylation in intact cells, we generated HeLa cells that stably expressed Flag-Bcl-w (HeLa/Bcl-w). HeLa/Bcl-w cells were stimulated with insulin or 10% serum for 15 min, and protein extracts then immunoprecipitated using an anti-Flag antibody and blotted with an anti-phospho (Ser/Thr) Akt substrate antibody that recognizes the Akt substrate motif. We found that the phosphorylated band corresponding to Bcl-w immunoprecipitates upon stimulation with serum or insulin. These results taken together provide evidence that Bcl-w may be a substrate of Akt both in vitro and in intact cells (Figure 4B).

RETRACTED

In turn, to investigate whether Bcl-w overexpression regulates Akt kinase activity, HEK293 cells were co-transfected with Flag-Bcl-w and HA-tagged Gsk3β, one of the main Akt substrates. 48 hours after transfection, the cells were stimulated with insulin for 10 min, cellular extracts immunoprecipitated with an anti-HA antibody, and then immunoblotted with an antibody that recognizes the phosphorylated form of Gsk3β. We did not find a change in the extent of Gsk3β phosphorylation by overexpressing Bcl-w (Figure 4C). Therefore, Bcl-w binds to Akt and is a direct substrate of Akt; however, this binding does not alter the activity of Akt on other substrates.

### Role of Bcl-w/Akt interaction on cell death

Given that Bcl-w is an anti-apoptotic member of the Bcl-2-family, we investigated the role of Akt activity on this function. We first analyzed the effect of Bcl-w overexpression in preventing apoptosis induced by two different chemotherapics, i.e. cisplatin and epirubicin, in HeLa/Bcl-w compared to parental untransfected HeLa cells. Cells were treated with 30 µg/ml cisplatin or with 10 µg/ml epirubicin for 24 hr. Cell death was assessed with a cell viability assay, with propidium iodide staining followed by FACS analysis, or by caspase 9, −3, and PARP activation. We found that HeLa/Bcl-w cells were 80–90% resistant to cell death induced by the chemotherapics. This was confirmed by analysis of the activation state of the intrinsic apoptotic pathway (caspase 9, −3, and PARP) (Figure 5A).

**Figure 5:** Akt regulates the anti-apoptotic function of Bcl-w. (A) HeLa control cells and HeLa cells stably expressing Flag-Bcl-w were plated in 96 well plates in triplicate and treated with 30 µg/ml of cisplatin or 10 µg/ml of epirubicin for 24 hr. Apoptosis was analyzed by Cell Vitality assay, by propidium iodide staining and FACS analysis, or by western blot for caspase cascade activation with anti-caspase-3, -9, and PARP antibodies. Loading control was obtained with anti β-actin. (B) HeLa-Flag Bcl-w cells were transfected with 4 µg of HA-Akt D− cDNA or with 100 nM of siAkt-RNA for 48 hrs and then treated with 30 µg/ml of cisplatin for 24 hr. Cell death was then analyzed as described above. Total lysates were analyzed by western blot using an anti-PARP antibody. Loading control was obtained with an anti-β-actin antibody. Inactivation of Akt activity resulted in a reduction in the protective effect of Bcl-w on cell death.

RETRACTED

To test the role of Akt activity on the antiapoptotic function of Bcl-w, we repeated the above experiments in Bcl-w/HeLa cells transfected for 48 hr either with Akt D− cDNA or with Akt siRNAs. We found that the inhibition of Akt kinase activity or protein quantity resulted in a strong activation of the downstream effector PARP (Figure 5 b, left panel), that is partially reflected as reduction of pro-survival effect of Bcl-w (∼20%) (Figure 5B). Thus, Akt activity mediates the anti-apoptotic function at least in part by regulating the intracellular levels of Bcl-w. Given that inhibiting Akt results in a reduction of Bcl-w levels, these results suggest that Akt may contribute to Bcl-w protective effects mainly by regulating its intracellular levels.

To further confirm this, we down-regulated Bcl-w expression with two specific Bcl-w-siRNAs, and analyzed the effects of Bcl-w down-regulation on chemotherapy-induced cell death. We found that 72 hrs of incubation with Bcl-w siRNAs drastically reduced Bcl-w protein (Figure 6 A) although to different extents (siRNA61 was more effective than siRNA62). The assessment of cell viability (Figure 6B) and of apoptotic cells (Figure 6C) provided evidence that the effect of cell death induced by chemotherapics was proportional to the expression of Bcl-w. Furthermore, by reducing Bcl-w level, we obtained the same ∼20% increase in cell death that we observed in HeLa cells treated with Akt siRNA. Thus, the reduction in Bcl-w expression secondary to Akt inactivation contributes to the resistance of cancer cells to chemotherapy-induced cell death.

**Figure 6:** Effects of Bcl-w si RNA on cell death. (A) Cells were transfected with 150 nM of siBcl-w-RNAs for 72 hrs. Total lysates were analyzed by western blot using anti-Bcl-w antibodies. Loading control was obtained with an anti-β-actin antibody. (B, C) Cells were transfected with 150 nM of siBcl-w-RNAs for 48 hrs. Then, the cells were splitted into 96 wells and then treated with 30 µg/ml of cisplatin for 24 hr. Cell death was then analyzed with MTT (B) or propidium iodide staining and FACS analysis (C). Bcl-w down-regulation induces an increase of cell death.

### Akt regulates Bcl-w interaction with Bcl-2 family members

The intrinsic apoptotic pathway is regulated by the net interactions of pro- and anti-apoptotic Bcl-2 members [22]. To evaluate the effect of Akt activity on the interaction of Bcl-w with the pro-apoptotic Bcl-2 members, we set up co-immunoprecipitation experiments with Bcl-w and Bad, Bik, or Bax in cells overexpressing the dominant negative Akt cDNA. We found that Akt inactivation resulted in a drastic reduction of Bcl-w interaction with the pro-apoptotic proteins (Figure 7). This further confirms the stimulatory role of Akt activity on Bcl-w anti-apoptotic function.

RETRACTED

**Figure 7:** (A) Akt activity regulates Bcl-w interaction with Bcl-2 family members. Flag-Bcl-w/HeLa cells were transfected with 2 µg of either HA-Akt D+ or HA-Akt D− cDNA, and 2 µg of EE-Bax cDNA for 48 hr. Cells were harvested and 1 mg of total lysate immunoprecipitated using an anti-Flag antibody. The immunoprecipitates were then blotted with an anti-EE antibody. Total protein was normalized using anti-EE, -HA or -β-actin antibodies, as indicated. (B) Flag Bcl-w/HeLa cells were transfected with 2 µg of HA-Akt D+ or HA-Akt D− cDNA, and 2 µg of either EE-Bad or EE-Bik cDNA, as indicated, for 48 hr. Cells were harvested and 1 mg of total lysate immunoprecipitated using anti-Flag antibody. The immunoprecipitates were then blotted with an anti-EE antibody. Total protein was normalized using anti-EE, -HA or -β-actin antibodies, as indicated. Inactivation of Akt induced a reduction of Bcl-w interaction with the pro-apoptotic Bcl-2 members.

## Discussion

Apoptosis is believed to be the major mechanism of chemotherapy-induced cell death in cancer [23], [24]. Unfortunately, many tumour cells evade drug-induced death signals [25]. Akt is an important survival-signaling molecule, whose function is frequently found altered in human cancer [5], [26]. Therefore, we decided to address the role of Akt in apoptosis resistance in human cancer by finding new partners of Akt by two hybrid screening in yeast. Among the interactors of Akt that we found, we focused on Bcl-w, a pro-survival member of the Bcl-2 protein family [27], [28] that has received less attention compared to its other family members. By genetic and biochemical methods, we have demonstrated here that Akt interacts with the N- and C-terminal sequences of the Bcl-w protein, and phosphorylates Bcl-w both in vitro and in the intact cell. The analysis of the Bcl-w sequence did not reveal a canonical Akt phosphorylation motif [29]. However, there is evidence that Akt may phosphorylate cellular substrates at the level of a partially conserved sequence motif [29]. Bcl-w posses at least 6 serine/threonines that are included in “degenerated” Akt phosphorylation sites. By site-directed mutagenesis, we mutated two of these sites (ser 62 and ser 83) substituting the serine with an alanine (data not shown). These mutations did not result in a change of Bcl-w phosphorylation state, so the hypothetical Akt phosphorylation site must be located elsewhere. We are now addressing this issue.

RETRACTED

We have also demonstrated here that interfering with the activity or amount of Akt reduces the quantity of Bcl-w protein; oppositely, transfection of a dominant active Akt mutant increased the content of Bcl-w in cells.

Akt-mediated Bcl-w down-regulation was observed to occur also in glioma (data not shown). Thus, Akt affects Bcl-w function in various cell types at least in part by regulating its expression. The mechanisms underlying this are not clear, but the regulation of Bcl-w protein levels is unlikely mediated by the ubiquitin-proteasome pathway, as evidenced by the negative result obtained with a proteasome inhibitor. Furthermore, Akt inhibition did not produce an effect on Bcl-w mRNA, as evaluated by Real Time PCR (data not shown). Other possible Akt-mediated regulatory effects on RNA or protein stability are under investigation in our laboratory.

Several studies have suggested that Akt may regulate the balance between pro- and anti-apoptotic signals, at least in part by regulating the cellular localization of Bcl-2 family members [30], [31]. Thus, in this study we have analyzed the effect of Akt activation on the subcellular localization of Bcl-w. We found Bcl-w predominantly associated with the mitochondrial fraction, as previously described also by O'Reilly et al. [32]. The presence of the kinase-dead Akt mutant reduced the amount of Bcl-w linked to this fraction, but it did not increase Bcl-w in the cytosol; we obtained similar results with cells transfected with Akt siRNA. Thus, via binding and phosphorylating Bcl-w, Akt may control Bcl-w activity mainly through the regulation of Bcl-w protein expression. We are conducting experiments with Bcl-w phosphorylation mutants to formally prove this conclusion.

Moreover, with the intent to clarify the role of Akt-mediated regulation of Bcl-w on its anti-apoptotic functions, we established a Bcl-w overexpressing cell line. These cells exhibit a significant decrease of chemotherapy-mediated cell death. When we evaluated the effects of decreasing Akt activity on survival in Bcl-w/HeLa cells, we found a ∼20% increase in cell death. However, when we analyzed cell death by western blot of PARP activation, the active PARP fragment was present exclusively in Bcl-w/HeLa cells incubated with Akt D− cDNA. Thus, even though the differences that we observe with FACS analysis and cell vitality are of small entity, the end point, that is cell death evaluated as PARP activation, is reached only in Bcl-w cells where Akt has been inactivated.

RETRACTED

On the other hand, our data provide evidence that Bcl-w is not the only defense mechanism of the cell toward chemotherapy-induced apoptosis, and many other Bcl-2 family members may mediate anti-apoptotic signals. Therefore, downregulation of Akt may result in a pronounced efficacy in cancer cells were Bcl-w predominates over the other Bcl-2 family members [33]–[35].

When appropriate stimuli are present, homodimerization of pro-apoptotic members of the Bcl-2 family activates the intrinsic apoptotic cascade. Bcl-w interacts with pro-apoptotic members of the Bcl-2 family, such as Bad, Bax, and Bik, blocking the formation of the homodimers and, thus, the activation of the apoptotic cascade. Events that inhibit the formation of these Bcl-w/pro-apoptotic Bcl-2 member complexes may lead to the activation of apoptosis [36]. We show here that Bcl-w/Bax, Bcl-w/Bad, and Bcl-w/Bik interactions were drastically reduced in cells overexpressing dominant-inactive Akt cDNA, indicating that Akt activity is necessary for these interactions. Therefore, Akt may regulate the anti-apoptotic function of Bcl-w, reducing its amount in the cell and, thus, impairing the balance of homo- and heterodimer formation upon apoptotic stimuli.

Bcl-w can be up-regulated in tumors such as gastric and colorectal cancer [33]–[35]. Interestingly, the PI3k-Akt pathway is involved in the progression and chemoresistance of these types of cancer [37]–[39]. Therefore, increased Akt activity can be speculated to promote survival and anti-apoptotic signaling in cancer cells at least in part through increasing Bcl-w levels. Recently, Bcl-w was reported to promote gastric cancer cell invasion, by inducing matrix metalloproteinase-2 expression [34]. Bcl-w is up-regulated also through pathways besides the Akt one: Tran et al. demonstrated that Bcl-w can be up-regulated via the NFkB pathway activated by TWEAK (tumor necrosis factor-like weak inducer of apoptosis) through stimulation of its receptor, Fn14; moreover, the TWEAK-Fn14 pathway can induce survival of glioma cells, at least in part by up-regulating the quantity of Bcl-w protein [40]. In addition, Yao et al. reported that up-regulation of Bcl-w protein mediates the neuroprotective effect of estrogens [41]. Therefore, Bcl-w participates in a number of different systems that regulate survival and anti-apoptotic pathways.

The results that we have presented here provide the first evidence that Akt interacts with, and regulates the levels of, Bcl-w, moving the balance of the Bcl-2 family toward anti-apoptotic members. Enhancement of this Akt/Bcl-w anti-apoptotic pathway can be speculated as one mechanism responsible for the reduced sensitivity to apoptosis of cancer cells that are resistant to chemotherapy-induced cell death. This finding may be of importance in optimizing a strategy for the treatment of cancers, such as gastric and colon adenocarcinoma, in which Bcl-w has been found to be increased.
